# LncRNA HAND2-AS1 exerts anti-oncogenic effects on bladder cancer via restoration of RARB as a sponge of microRNA-146

This article has been retracted.

**DOI:** 10.1186/s12935-021-02063-y

**Published:** 2021-07-08

**Authors:** Liping Shan, Wei Liu, Yunhong Zhan

**Affiliations:** 1 Department of Urology, Shengjing Hospital, China Medical University, 36 Sanhao Street, Heping District, Shenyang, 110004 Liaoning China; 2 Emergency Department, First Hospital of China Medical University, Shenyang, Liaoning China

## Abstract

**Background:**

Growing evidence has shown that long noncoding RNA: microRNA: mRNA is implicated in tumor initiation, development, and progression. Long noncoding RNA HAND2-AS1 exhibits anti-cancer effects in diverse cancers. However, the knowledge of HAND-AS1 in bladder cancer development remains unknown.

**Methods:**

LncRNA and miRNA microarray was conducted to explore different expressed RNA in primary bladder cancer specimens. RNA-RNA interaction prediction tools miRcode (http://www.mircode.org/), DIANA-lncBase v2 (https://carolina.imis.athena-innovation.gr/diana_tools/web/index.php?r=lncbasev2%2Findex-experimental), DIANA-TarBase v.8 (https://carolina.imis.athena-innovation.gr/diana_tools/web/index.php?r=tarbasev8%2Findex) and miRDB (http://www.mirdb.org/) were employed to predict the interactions between RNA. Bladder cancer cell lines were used to perform cell proliferation and apoptosis assays. Western blot and quantitative Real-time Polymerase Chain Reaction were used to determine the expression of protein and RNA separately. Dual-luciferase assay was conducted to determine the activity of three prime untranslated region of retinoic acid receptor beta (RARB). Furthermore, 5637 human bladder cancer mouse models were established to investigate the interactions of lncRNA: miRNA: mRNA in vivo.

**Results:**

Based on the RT2 lncRNA PCR Arrays analysis, we validated HAND2-AS1 declined in bladder cancer and negatively correlated with the depth of invasion and grades. The overexpression of HAND2-AS1 in human bladder cancer cells 5637 and RT4 hampered cell proliferation by provoking Caspase 3-triggered cell apoptosis. Besides, one of the HAND2-AS1 sponges, miR-146, elevated in bladder cancer and targeted the tumor suppressor, retinoic acid receptor beta (RARB). We further demonstrated that the HAND2-AS1: miR-146: RARB complex promoted Caspase 3-mediated apoptosis by suppressing COX-2 expression. Finally, the results gained in mouse xenografts suggested that HAND2-AS1 diminished miR-146 expression, thereby reversing the suppression of miR-146 on RARB-mediated apoptosis and contributing to bladder cancer regression.

**Conclusion:**

The present study sheds light on the fact that lncRNA HAND2-AS1 exerted as a tumor suppressor by releasing RARB from miR-146, leading to tumor proliferation and invasion inhibition. The findings expanded HAND2-AS-mediated regulatory networks' knowledge and provided novel insights to improve the RARB-targeted regimens against bladder cancer.

**Supplementary Information:**

The online version contains supplementary material available at 10.1186/s12935-021-02063-y.

## Background

In the light of National Central Cancer Registry of China 2015 annual report, bladder cancer is the sixth most common cancer in males and 15th in females [1]. The estimated mortality of bladder cancer was 25,100 and 7800 for men and women, separately. Although a declined mortality was gain in the last analysis, the bladder cancer burden in China will probably elevate in the coming decades due to population aging and environmental pollution, such as tobacco consumption [2]. Because the treatment mainly determines mortality, the improvement of clinical outcomes, including targeted therapy and immunotherapy against advanced bladder cancer, is imperative.

Abnormal expression of noncoding RNAs, including long-noncoding RNA (lncRNA) and micro-RNAs (miRNAs), are found frequently in carcinogenesis [3]. The mature noncoding RNAs do not translate to protein, whereas they regulate gene expression in various styles [4, 5]. Particularly, lncRNA binds to the single strand mRNA, hampering the translation into protein of target genes or resulting in mRNA degradation [6]. Furthermore, lncRNAs serve as a molecular decoy, sponge miRNA, and interrupt the association of miRNAs and messenger RNAs (mRNA). Besides, lncRNAs are involved in epigenetic- and post-transcriptional regulation of multiple genes, contributing to bladder cancer malignancy development [7]. Although a tremendous amount of lncRNA has been clarified, much remains unknown about the roles of lncRNA involving the progression of bladder cancer.

miRNAs are small noncoding RNAs that regulate cancer initiation, proliferation, migration, angiogenesis, and drug resistance by targeting mRNAs [8, 9]. For example, miR-205 inhibited cell proliferation via targeting cyclin J [10]. miR-96 provoked proliferation and antagonized apoptosis by targeting the cyclin-dependent kinase inhibitor 1A, CDKN1A [11]. Besides, multiple studies indicated miRNAs interacted with lncRNA, modulated the transcriptome further [12]. To fully understand lncRNA's tasks in regulating bladder cancer progress, investigating the complex network between lncRNA: miRNAs: mRNAs is fundamental.

In the present study, we aimed to shed light on the expression of HAND-AS1, miR-146, and retinoic acid receptor-β in bladder cancer by employing clinical samples and cell lines. Moreover, we attempted to evaluate the interplay of lncRNA, miRNA, and mRNA in bladder cancer progression and the mechanisms in malignancy by conducting knockdown- and rescue experiments.

## Methods

### Patients and specimens

Thirty-two patients who had primary bladder cancer were recruited at Shengjing Hospital of China Medical University from 2013 to 2018. Patients who received pre- or postoperative chemotherapies or targeted therapies were excluded. The study was approved by the Medical Ethics Committee of Shengjing Hospital of China Medical University. All participants provided written informed consent for research purposes and publications. Patients with an average age of 55.63 years (range from 42 to 81 years). Two independent pathologists reviewed all patients' slides to validate the diagnosis and to classify the tumor according to TNM Stage. 13 patients were diagnosed as T1, 9 patients were diagnosed as T2, 8 patients were diagnosed as T3, and 2 patients were diagnosed as T4. Adjacent tissues and tumor tissues were collected simultaneously. All specimens were placed immediately into liquid nitrogen and stored at − 80 °C.

### LncRNA and miRNA microarray analysis

Total RNA from bladder cancer and adjacent tissues were analyzed with RT^2^ lncRNA PCR Arrays and miRNA qPCR Assay (QIAGEN NV Corporate, Venlo, The Netherlands). Microarray analysis was performed with the Data Analysis Center as previously described [13]. Data obtained from three independent experiments and RNAs (fold change > 1.5 and P-values < 0.05) were considered expressed differentially between the two groups. All data has been curated by the Gene Expression Omnibus database, and the accession number is GSE140584, GSE140585 and GSE140587.

### Discovery of lncRNA-miRNA-mRNA associations

Interactions between lncRNA and miRNA were predicted with miRcode, and DIANA-lncBase v.2 followed the previously described [14, 15]. Connections between miRNA and mRNA were predicted with DIANA-TarBase v.8 [16] and miRDB [17].

### Cell culture, transfection reagents, and antibodies

Human SV40 immortalized uroepithelium cell SV-HUC-1 (CRL-9520™), Human urinary bladder cell lines 5637 (HTB-9™), RT4 (HTB-4™) and J82 (HTB-1™) were purchased from American Type Culture Collection (ATCC, Manassas, VA, USA). Cells were maintained in Dulbecco's modified Eagle medium with 10% fetal bovine serum (Thermo Fisher Scientific Inc., Waltham, MA, USA) at 37^◦^C and 5% CO_2._ Vendors have claimed that cells have been tested for mycoplasma contamination regularly.

Control vector pDonor-SH01 (SH025), HAND2-AS1 (DC-W1888-SH01), RARB (A0018), Scrambled control (CSHCTR001-CH1), sh-RARB (HSH070504-CH1) were purchased from GeneCopoeia, Inc. (Rockville, MD, USA). si-negative control, si-HAND2-AS1, Scrambled-miR Control, miR-146 mimic, miR-146 inhibitor, and miR-146 mutant were synthesized by GenePharma Co., Ltd. (Shanghai, China). Antibodies against RARB (sc-514585), COX-2 (sc-376861), Caspase 3 (sc-7272), and GAPDH (sc-47724) were obtained from Santa Cruz Biotechnology, Inc (Dallas, Texas, USA).

### Cell proliferation analysis

5 × 10^3^ 5637 or RT4 cells/well were allowed to attach 96-well plates overnight, and 20 μl of a 5 mg/ml stock of methylthiazolyldiphenyl-tetrazolium bromide (MTT, 298–93-1, Sigma-Aldrich Inc., St. Louis, MO, USA) was added to the medium post-treatment for 0, 12, 24, 36, or 48 h. After four hours, the supernatant was discarded, and the pellet was dissolved in 150 μl of Dimethyl Sulfoxide (CAS 67-68-5, Santa Cruz Biotechnology, Inc. Dallas, Texas, USA). A microplate reader (Bio-Rad 680 XR, Hercules, CA, USA) was used to detect the absorbance at 490 nm.

### Apoptosis analysis

1.5 × 10^5^ cells per well were seeded in 6-well plates. After 12 h, experimental treatments were performed. Cells were stained with the ANNEXIN V-PI (sc-4252 AK, Santa Cruz Biotechnology, Inc. Dallas, Texas, USA) followed the manufacture's instructions. The fluorescence in thrice independent experiments were determined by flow cytometry.

### Western blot

Tissues and cells were washed twice with pre-cooled PBS and lysed with lysis buffer for 30 min on ice. The concentrations of protein content were determined using a BCA protein assay kit (23225, Pierce; Thermo Fisher Scientific Inc., Waltham, MA, USA). Equal amounts of 25 µg proteins were resolved by 10% SDS-PAGE and transferred onto polyvinylidene fluoride membranes. The membranes were blocked with 5% skim milk in TBS-T for one h at room temperature and incubated with specific primary antibodies (1:1000) at 4 °C with gentle shaking overnight. Membranes were washed three times with TBS-T following incubation with secondary antibodies conjugated to HRP (1:2500; CatLog 31430 and CatLog 31460, Thermo Fisher Scientific Inc., Waltham, MA, USA). The complexes of antibody: protein was detected by enhanced chemiluminescence (Pierce; Thermo Fisher Scientific Inc., Waltham, MA, USA).

### Quantitative real-time polymerase chain reaction (qRT-PCR)

Total RNA was extracted by 1 ml TRIzol (Merck & Co., Inc., Kenilworth, NJ, USA) adapted to the manufacturer's protocol. 500 µg RNA was reverse transcribed to cDNA in 20 μl system by First Strand cDNA Synthesis Kit for RT-PCR (Merck & Co., Inc., Kenilworth, NJ, USA). Real-time PCR was performed using the Mx3000P real-time PCR system (Thermo Fisher Scientific, Waltham, MA, USA). PCR was carried out as follows: 40 cycles of 94 °C for 15 s, 60 °C for 10 s, and 72 °C for 20 s. All procedures were performed independently three times. Gene expression was normalized to the GAPDH to calculate relative expression using the 2^−ΔΔCq^ method [18]. The primer sequences used in this study were listed as below: HAND2-AS1, forward: 5′-GGGTGTTTACGTAGACCAGAACC-3′; reverse: 5′-CTTCCAAAAGCCTTCTGCCTTAG-3′; *GAPDH*: forward:5′-GTCTCCTCTGACTTCAACAGCG-3′; reverse: 5′-ACCACCCTGTTGCTGTAGCCAA-3′; miR-146: forward: 5′-GAGAACTGAATTCCATGG-3′; reverse: 5′-GAACATGTCTGCGTATCTC-3′; *U6*: forward: 5′-CGAGCACAGAATCGCTTCA-3′; reverse: 5′-CTCGCTTCGGCAGCACATAT-3′; *RARB*, forward: 5′-GGTTTCACTGGCTTGACCATCG-3′; reverse: 5′-CCGTCTGAGAAAGTCATGGTGTC-3′; *COX-2*, forward: 5′-CGGTGAAACTCTGGCTAGACAG-3′; reverse: 5′-GCAAACCGTAGATGCTCAGGGA-3′; *Caspase 3,* forward: 5′-TGGCCCTGAAATACGAAGTC-3′; reverse: 5′-GGCAGTAGTCGACTCTGAAG-3′.

### Dual-luciferase reporter assay

Dual-luciferase activity assay was performed as described previously [19]. The RARB or RARB Mut 3′-UTR was amplified and inserted into the pMIR-REPORTTM vector (Thermo Fisher Scientific, Waltham, MA, USA) followed the manufacturer's direction. 1 × 10^4^ cells were plated in a 96-well plate and were allowed to attach overnight. miR-146 mimic or scrambled-miR control was transfected into cells combined with 100 ng of RARB or RARB Mut 3′-UTR. Luciferase activity was determined with the dual-luciferase reporter assay system post-24 h transfection with the Luciferase Reporter Assay System (Promega, Madison, WI, USA). Renilla luciferase was used as an internal control in the Luciferase Reporter Assay according to the vendor's protocol.

### Immunohistochemical staining

Expression of RARB in formalin-fixed, paraffin-embedded tissues were detected by anti-RARB (sc-514585) at a dilution of 1:100. Antigen was retrieved after heating in pH 6.0 citrate buffer. Slides then were incubated with streptavidin–horseradish peroxidase-conjugated secondary antibodies (Maixin, Fuzhou, China) according to the vendor’s instructions.

### Generation of 5637 human bladder cancer mouse models

All studies that involved experimental animals were approved by the medical ethics committee of Shengjing Hospital of China Medical University and conducted according to the guidelines of the center of experimental animals of Shengjing Hospital of China Medical University. Female BABL/c athymic nude mice (five-week-old) were obtained from Beijing Vital River Laboratory Animal Technology Co., Ltd (Beijing, China) and housed under specific-pathogen-free conditions. Cells expressing HAND2-AS1, miR-146, or vector stably were subcutaneously injected into the right flanks of mice. Eighteen mice that harbored approximately 100 mm^3^ tumors were divided into three groups randomly (six per group) from day 0. The tumor volumes were measured and recorded every four days. Twenty-eight days later, all mice were euthanized, and tumors were resected, fixed, and weighed.

### Statistical analysis

The data from all experiments were presented as means plus standard deviation. The association between lncRNA HAND2-AS1 and miR-146 expression was analyzed by Spearman's correlation coefficient. Kaplan–Meier survival analysis was used to estimate the correlation of HAND2-AS1 expression and survival times of bladder cancer. The differences in groups were evaluated by One Way Analysis of Variance (ANOVA) with LSD test or by Two-way ANOVA with Tukey's multiple comparisons test. *P* < 0.05 indicated by '*' or '#' respectively were statistically significant. Statistical analysis was conducted using GraphPad version 7.0 (San Diego, CA, USA).

## Results

### LncRNA HAND2-AS1 expression decreases in bladder cancer and correlated with more prolonged overall survival

Ten LncRNA was verified to express differentially in bladder cancer specimens, among which the difference in HAND2-AS1 was the most significant (Fig. 1A). To confirm the distinctly expressed lncRNA HAND2-AS1, we employed qRT-PCR analysis. Consistent with the result in Fig. 1A, HAND2-AS1 expression declined evidently in bladder cancer compared to paired adjacent tissues (1.29 vs. 2.004, *P* < 0.01, Fig. 1B). The HAND2-AS1 expression was further evaluated in cell lines. As shown in Fig. 1C, RT4 cells had the highest expression of HAND2-AS1 while 5637 and J82 cells expressed equal HAND2-AS1. Therefore, we selected 5637 and RT4 cells for the following experiments. Moreover, we attempted to reveal the relationship between HAND2-AS1 expression and survival time. According to the expression value of each patient, we classified patients into two categories and detected their prognosis. We analyzed the prognosis of each category of patients by Kaplan–Meier survival estimators, followed by log-rank tests. We determined all values between 20 to 80th percentiles to choose the best cut-offs for categorizing patients in the survival outcomes. The significant differences in the groups and the value emerging the lowest log-rank P value was selected. Figure 1D showed the patients with higher HAND2-AS1 expression had a longer overall survival time. Additionally, Table 1 summarized the HAND2-AS1 expression related to grades (*P* = 0.0309) and invasive depth (*P* = 0.0074) of bladder cancer, suggesting that HAND2-AS1 played a pivotal role in bladder cancer. No significant connection was found between HAND2-AS1 expression and gender, ages, tumor size, nodes, metastasis, or stages. Collectively, these results indicated that HAND2-AS1 was involved in bladder cancer progression.

**Fig. 1:** LncRNA HAND2-AS1 expression declines in bladder cancer and correlates with more prolonged overall survival. **A** Differential lncRNA expression in bladder cancer was analyzed by RT^2^ PCR array. Data obtained from triple paired bladder cancer tissues and adjacent tissues. The color indicated the fold change of target gene normalized to housekeeping genes. **B** HAND2-AS1 expression was reduced in bladder cancer tissues. **P < 0.01, vs. adjacent tissues, n = 32. **C** HAND2-AS1 expression declined in bladder cancer cell lines. *P < 0.05, vs. SV-HUC-1, n = 3. **D** The association of HAND2-AS1 expression and overall survival of bladder cancer

**Table 1:** The relationship between HAND2-AS1 expression and clinical characteristics of bladder cancer

Variables	Description	No. of patient	HAND2-AS1 expression		χ^2^	*P*-value
			Low	High		
Gender	Male	22	16	6	0.0253	0.873
	Female	10	7	3		
Age (years)	< 60	8	6	2	0.0515	0.820
	≥ 60	24	17	7		
Tumor size	≤ 3 mm	10	5	5	3.4431	0.063
	> 3 mm	22	18	4		
Depth of invasion	Tis-T1	13	6	7	7.1656	0.007*
	T2–T4	19	17	2		
Nodes	N0	18	8	10	1.24494	0.264
	N1–N3	14	9	5		
Metastasis	M0	21	12	9	0.396028	0.529
	M1	11	5	6		
Grades	G1	9	4	5	4.6608	0.030*
	G2–G3	23	19	4		
Stages	Stage 0–2	13	9	10	0.9579	0.327
	Stage 3–4	19	12	7		

*T* tumor, *N* nodes, *M* metastasis, *G* grades

* *P* < 0.05 was statistically significant

### LncRNA HAND2-AS1 inhibits cell proliferation by promoting apoptosis

Based on the result that the reduction of HAND2‐AS1 predicted shorter overall survival than the increment of HAND2-AS1, we determined the proliferation of cells expressing HAND2-AS1 or si-HAND2-AS1 by MTT assay. Figure 2A showed that overexpression of HAND2-AS1 suppressed cell proliferation notably, whereas impairment of HAND2-AS1 by si-RNA triggered cell proliferation (Fig. 2B). Results in 5637 and RT4 cells were identical. To investigate the effects of HAND2-AS1 on apoptosis, we carried out Annexin-V FITC fluorescence analysis. The results in Fig. 2C indicated that HAND2-AS1 enhanced 5637 apoptosis (5.98% vs. 1.61%, *P* < 0.05) while si-HAND2-AS1 repressed apoptosis (0.63% vs. 1.40%, *P* < 0.05) compared to the respective control (Fig. 2D). These results suggested that overexpression of HAND2-AS1 inhibited cell proliferation and enhanced apoptosis.

**Fig. 2:** The overexpression of lncRNA HAND2-AS1 inhibits cell proliferation by promoting apoptosis. MTT assay was performed with cells post introduction of HAND2-AS1 (**A**) or si-HAND2-AS1 (**B**). *P < 0.05, n = 3. FITC-PI apoptosis analysis was performed with cells post-introductions of HAND2-AS1 (**C**) or si-HAND2-AS1 (**D**). Representative images of flow cytometry were shown. Data obtained from three independent experiments. *P < 0.05, vs. vector or si-NC. si-NC, silence negative control RNA

### LncRNA HAND2-AS1 serves as the sponge of miR-146

miRNA array analysis revealed that miR-146 (alias for miR-146a-5p) enriched in bladder cancer (Additional file 1: Table S1); therefore, we attempted to explore miR-146 in the following study. The further investigation evaluated the miR-146 expression elevated in bladder cancer tissue compared to adjacent tissue (1.685 vs. 0.791, *P* < 0.05, Fig. 3A). We detected the expression of miR-146 in uroepithelium cell SV-HUC-1, bladder cancer cells 5637, RT4, and J82. Figure 3B showed that miR-146 elevated in bladder cancer cells compared to SV-HUC-1. The expression of miR-146 in 5637 was higher than that in RT4, while miR-146 expression in J82 was similar to 5637. More importantly, miR-146 expression was related to HAND2-AS1 negatively (*P* = 0.0047, Fig. 3C), indicating that HAND2-AS1 sponged miR-146 in bladder cancer cells and deregulated miR-146 expression. According to the predicted association by miRcode11, the putative binding sites located in chromasome4: 174,461,274–174,461,279 and chromasome4: 174,506,582–174,506,586 (http://mircode.org/?gene=ENSG00000237125&mirfam=miR-146&class=lncRNA&cons=&trregion=). We hence generated miR-146 mutant (miR-146MUT), where the potential sponge sites were disrupted (Fig. 3D). As expected, the relative expression of miR-146WT (miR-146 mimic) fell apparently in cells overexpressing HAND2-AS1, while that increased in HAND2-AS1-knockdown cells (Fig. 3E). The expression of miR-146MUT changed hardly in cells post introduction of HAND2-AS1 or si-HAND2-AS1 compared to the corresponding control group, implying HAND2-AS1 had little effect miR-146MUT. The results demonstrated that HAND2-AS1 sponged miR-146 and inhibited miR-146 expression.

**Fig. 3:** LncRNA HAND2-AS1 functions as a sponge for miR-146. **A** miR-146 expression in bladder cancer specimens was determined by qRT-PCR. *P < 0.01, vs. adjacent tissues, n = 32. **B** miR-146 expression in the indicated cell lines was determined by qRT-PCR. *P < 0.05, n = 3. **C** The correlation of miR-146 and HAND2-AS1 expression. n = 32. **D** Schematic diagram of the putative binding sites of HAND2-AS1 and miR-146. **E** The relative activity of the miR-146 promoter in the indicated cells was determined by dual-luciferase assay. miR-146wt, miR-146 wild-type promoter. miR-146mut, miR-146 mutated promoter. *P < 0.05, vs. control, n = 3. #*P* < 0.05, vs. si-NC, n = 3. **F** The expression of miR-146 wt or miR-146mut in 5637 cells expressing HAND2-AS1 or si-HAND2-AS1 was accessed by qRT-PCR. *P < 0.05, vs. control, n = 3. #*P* < 0.05, vs. si-NC, n = 3

### miR-146 triggers cell proliferation by targeting RARB

To detect the target genes of miR-146, we used prediction algorithms such as DIANA-TarBase (http://carolina.imis.athena-innovation.gr/diana_tools/web/index.php?r=tarbasev8%2Findex) and miRDB (http://mirdb.org/index.html). We found that the expression of retinoic acid receptor beta (RARB) was decreased in cancer samples compared to adjacent samples (Fig. 4A, B). Besides, RARB expression was positively related to HAND2-AS1 (Fig. 4C); hence, we selected RARB for further exploring among the several candidate target genes. To validate the effects of potential binding sites on miR-146: RARB complex, we produced mutated RARB 3'UTR (RARB Mut), which lacked binding capacity (Fig. 4D). We confirmed that miR-146 mimics repressed the relative activity of RARB 3'UTR significantly, while miR-146 inhibitor trigged the activity by dual-luciferase assay. Nevertheless, miR-146 mimics or miR-146 inhibitor hardly changed the activity of mutated RARB 3'UTR compared to the scrambled RNA (Fig. 4D). To confirm the suppression of RARB by miR-146, we conducted qRT-PCR assays. As shown in Fig. 4E, miR-146 mimics inhibited RARB expression, whereas miR-146 inhibitor enhanced RARB expression in comparison with scrambled RNA in 5637 cells. The transfection efficiency of miR-146 was validated as well. Identical results were observed in RT4 cells. Furthermore, the RARB expression increased notably in cells expressing HAND2-AS1, while that decreased in cells lacking HAND2-AS1, consistent with the alteration in RNA levels (Fig. 4F). To estimate the effects of miR-146 on cell proliferation, we performed MTT assay further. Figure 4G showed that cell proliferation increased by sh-RARB while that dropped by miR-146 inhibitor. Notably, the combination of miR-146 inhibitor and sh-RARB diminished miR-146 inhibitor-enhanced proliferation. These results suggested that miR-146 targeted RARB directly and promoted cell proliferation via the downregulation of RARB.

**Fig. 4:** The overexpression of miR-146 promotes cell proliferation by targeting RARB. **A**, **B** The expression of RARB in cancer tissues and the corresponding adjacent tissues was determined by immunohistochemical staining and qRT-PCR, respectively. *P < 0.05 vs. adjacent tissues. adj, adjacent tissues; can, cancer tissues. **C** The relationship between RARB and HAND2-AS1 expression in 32 pairs of bladder cancer tissues. **D** Left panel, schematic of the predicted binding sites of miR-146 and RARB; Right panel, the relative activity of the RARB promoter was determined by dual-luciferase assay. RARB, RARB wild type 3′-UTR; RARB Mut, RARB mutated 3′-UTR; miR-146 in, miR-146 inhibitor. **P < 0.01, vs. scramble RNA, n = 3. **E** The expression of RARB or miR-146 in the indicated cells was analyzed by qRT-PCR. *P < 0.05, vs. scrambled RNA, n = 3. Scr, scrambled RNA. **F** The expression of RARB in the indicated cells was analyzed by western blot. **G** The proliferation of 5637 and RT4 cells expressing miR-146in, sh-RARB or the combination was accessed by MTT assay. miR-146 in, miR-146 inhibitor. sh-RARB, shRNA targeting RARB. *P < 0.05, vs. control, n = 3. Scr, scramble RNA

### LncRNA HAND2-AS1 suppresses cell proliferation via releasing RARB from miR-146

To determine the effects of HAND2-AS1: miR-146: RARBs in cell proliferation, we conducted MTT assay. Figure 5A showed the ectopic expression of HAND2-AS1 repressed 5637 cell proliferation, while the combination of HAND2-AS1 and miR-146 mimics reversed the suppression. Identical results were obtained in RT4 cells. Moreover, Annexin-V fluorescence analysis was performed to determine the alteration of cell apoptosis. Figure 5B exhibited the representative images of flow cytometry analysis (left panel). The right panel of Fig. 5B showed that HAN2-AS1 triggered apoptosis of 5637 cells (1.76%), while miR-146 diminished that of 5637 cells (0.53%) compared to the control (0.80%). However, the co-expression of HAND2-AS1 and miR-146 hindered the deregulation of apoptosis by miR-146 (0.76% vs. 0.80%, *P* > 0.05). Likewise, overexpression of HAND2-AS1 and miR-146 simultaneously impaired the declined apoptotic RT4 cells (0.56% vs. 0.52%, *P* > 0.05). To investigate the connections among HAND2-AS1: miR-146: RARB, qRT-PCR, and western blot were performed. Figure 5C showed that RARB expression increased in cells expressing HAND2-AS1 accompanied by the increment of Caspase 3, the predominant executor of apoptosis. Conversely, the expression of RARB and Caspase 3 declined in cells expressing miR-146 compared to control. Furthermore, forced expression of HAND2-AS1 along with miR-146 overcame the HAND2-AS1-induced RARB expression. Similar results were obtained in RT4 cells. To further clarify the mechanisms underlying the association of HAND2-AS1: miR-146: RARB, we determined the expression of COX-2, a key regulator of producing prostaglandin E2 in cells 5637 and RT4. The results in Fig. 5D indicated RARB and Caspase 3 expression elevated, while that of COX-2 descended significantly by overexpression of HAND2-AS1. Inversely, the expression of RARB and Caspase 3 declined while that of COX-2 elevated evidently by overexpression of miR-146. Briefly, these results suggested that HAND2-AS1 repressed cell proliferation through hampering miR-146: RARB interaction.

**Fig. 5:** The overexpression of lncRNA HAND2-AS1 attenuates cell proliferation and enhances apoptosis by releasing RARB from miR-146. **A** The proliferation of the indicated cells was accessed by MTT assay. *P < 0.05, vs. control, n = 3. **B** The apoptosis of the indicated cells was detected by FITC-PI stain, followed by flow cytometry analysis. Representative images of three independent experiments were shown. *P < 0.05 vs. vector. ns, no significance. **C** The expression of HAND2-AS1, miR-146, RARB, and Caspase 3 in the indicated cells were measured by qRT-PCR. *P < 0.05 vs. control, n = 3. ns, no significance. **D** The expression of HAND2-AS1, miR-146, RARB, and Caspase 3 in the indicated cells were measured by western blot

### LncRNA HAND2-AS1 suppresses tumor growth in vivo

To illustrate if HAND2-AS1 inhibited tumor growth via miR-146: RARB in vivo, we established 5637 human bladder cancer mouse models. Cells expressing HAND2-AS1, miR-146 or vector stably were subcutaneously injected into nude mice. The tumor growth curves in Fig. 6A demonstrated that overexpression of HAND2-AS1 attenuated tumor growth significantly, while the co-expression of HAND2-AS1 and miR-146 overwhelmed the inhibition. The alteration of tumor weights was similar to that of tumor growth (Fig. 6B). Figure 6C exhibited the representative images of tumors in each group. The upregulation of HAND2-AS1 reduced tumor weights, whereas the combination conquered the inhibition completely. The overexpression of HAND2-AS1 enhanced RARB and Caspase 3 expression while repressing COX-2 expression (Fig. 6D). Besides, the changes of the RARB, COX-2, and Caspase 3 were comparable to those in protein levels (Fig. 6E). The results gained in the animal model suggested that the overexpression of miR-146 inhibited RARB expression and subsequently repressed RARB-mediated signaling cascades. The results indicated that HAND2-AS1 worked as a tumor suppressor by rescuing RARB from miR-146.

**Fig. 6:** The overexpression of lncRNA HAND2-AS1 suppresses tumor growth in 5637 human bladder cancer mouse models. **A** Tumor growth curves of xenografts for four weeks. *P < 0.05; ns, no significance, vs. vector, 6 mice per group. **B** The median weights of tumors per group. *P < 0.05; ns, no significance, vs. control, 6 mice per group. **C** The representative images of gross examination in each group were shown. **D** The expression of the indicated protein in tumor models was determined by western blot. **E** The expression of HAND2-AS1, miR-146, RARB, and Caspase 3 in tumors was determined by qRT-PCR. *P < 0.05 vs. control, n = 6

## Discussion

LncRNA heart and neural crest derivatives expressed 2-antisense RNA 1 (HAND2-AS1) was discovered for the first time in hepatocellular carcinoma. Luo and colleagues found that HAND2-AS1 expression dropped in hepatocellular carcinoma and was related to metastasis [20]. Growing evidence revealed that HAND2-AS1 suppressed tumor progression via multiple signaling pathways in various cancers, including endometrioid endometrial carcinoma [21, 22], head and neck squamous cell carcinoma [23], osteosarcoma [24, 25], colorectal cancer [26, 27], non-small cell lung cancer [28], esophagus squamous cell carcinoma [29], ovarian cancer [30], melanoma [31], and cervical squamous cell carcinoma [32]. Nevertheless, the role of HAND2-AS1 in bladder cancer progression is unclear yet. In the present study, we observed HAND2-AS1 expression was decreased in bladder cancer tissues compared to adjacent noncancerous tissues. Furthermore, we demonstrated that HAND2-AS1 expression was negatively correlated with the overall survival times of bladder cancer. Additionally, HAND2-AS1 expression was associated with invasive depth and differentiation significantly. These results implied that HAND2-AS1 served as a tumor suppressor in bladder cancer progression, which were concordant with the previous studies.

There are two members in the human miR-146 family, miR-146a (alias: miR-146) and miR-146b. These two miRNAs have similar sequences and share identical seed regions; however, they are located on different chromosomes and display diverse regulation in multiple biological functions by targeted various genes [33]. So far, four transcription factors were able to regulate miR-146 expression by cohering with the promoter region of miR-146, including the transcription factor nuclear factor κ-light-chain-enhancer of activated B cells [34], the interferon regulatory factor 3/7, the CCAAT-enhancer-binding-protein-β [35], and the Myc proto-oncogene protein [36]. We clarified that miR-146 combined with the transcript region of HAND2-AS1. The results suggested HAND2-AS1 bind to miR-146 and impeded the miR-146: RARB interaction as competitive endogenous RNA. Although supplementary experiments beyond bladder cancer are required, our findings enlarged the knowledge of the regulation network of miR-146.

Among the redundant targeted genes of miR-146, RARB expression was reduced significantly in bladder cancer. In the last decades, many studies have revealed that loss of RARB expression predicted progressive behavior in premalignant and malignant tissues, as well as the immortal cells [37]. Nevertheless, the mechanisms underlying the downregulation of RARB were not fully investigated. Xu has reviewed that several transcriptional factors and epigenetic mechanisms, such as histone deacetylation and methylation, contributed to the deregulation of RARB [38]. Particularly, the RAR-β2 promoter methylation was accessed as a biomarker to predict survival for multiple human cancer. Apart from the aforementioned factors, dozens of miRNAs have been demonstrated to suppress the RARB expression. RARB expression can be regulated by HAND2-AS1: miR-146 interaction, supplementing the knowledge about the deregulation of RARB. In addition to the regulation of RARB, we unveiled the alteration of COX-2 was opposite to RARB and Caspase 3 in vitro and in vivo. The results were in agreement with previous studies. During the process of human carcinogenesis, COX-2 served as a joint in the complex network where RARB inhibited COX-2 expression, leading to proliferation reduction [39–41]. COX-2 also antagonized Caspase 3-mediated apoptosis, conferring chemoresistance [42].

The numbers of clinical specimens in the current study are limited. Therefore, detecting HAND2-AS1 expression in clinical samples covering benign and malignancy, initial and advanced stages, primary and recurrent cases are necessary for drawing the global pictures of HAND2-AS1 regulation networks in bladder cancer. Moreover, the potential interaction of HAND2-AS1 and other signaling pathways convergent on RARB should be investigated carefully. Finally, the connection between transcriptive regulation and methylation of RARB cannot be ruled out.

## Conclusion

To summarize, our study identified that the lncRNA HAND2-AS1 expression was negatively correlated to poor clinical outcomes of bladder cancer. Furthermore, we confirmed that HAND2-AS1 suppressed cell proliferation by sponging miR-146 and rescuing RARB from miR-146 as a competitive endogenous RNA. Our findings extended the understanding of the interplay of HAND2-AS1/miR-146/RARB, which took part in regulating bladder cancer regression.

## Supplementary Information

**Additional file 1.** Additional table.

**Additional file 2: Fig. S1**. LncRNA HAND2-AS1 expression declines in bladder cancer and correlates with more prolonged overall survival. (**A**) Differential lncRNA expression was analyzed in bladder cancer by RT2 PCR array. Data obtained from triple paired bladder cancer tissues and adjacent tissues. The color indicated the fold change of target gene normalized to housekeeping genes. (**B**) HAND2-AS1 expression reduced in bladder cancer tissues. **P<0.01, vs. adjacent tissues, n=32. (**C**) HAND2-AS1 expression declined in bladder cancer cell lines. *P<0.05, vs. SV-HUC-1, n=3. (**D**) The association of HAND2-AS1 expression and overall survival of bladder cancer.

**Additional file 3: Fig. S2**. The overexpression of lncRNA HAND2-AS1 inhibits cell proliferation by promoting apoptosis. MTT assay was performed with cells post introduction of HAND2-AS1 (**A**) or si-HAND2-AS1 (**B**). *P<0.05, n=3. FITC-PI apoptosis analysis was performed with cells post-introductions of HAND2-AS1 (C) or si-HAND2-AS1 (D). Representative images of flow cytometry were shown. Data obtained from three independent experiments. *P<0.05, vs. vector or si-NC. si-NC, silence negative control RNA

**Additional file 4: Fig. S3.** LncRNA HAND2-AS1 functions as a sponge for miR-146. (**A**) miR-146 expression in bladder cancer specimens was determined by qRT-PCR. *P<0.01, vs. adjacent tissues, n=32. (**B**) miR-146 expression in the indicated cell lines was determined by qRT-PCR. *P<0.05, n=3. (**C**) The correlation of miR-146 and HAND2-AS1 expression. n=32. (**D**) Schematic diagram of the putative binding sites of HAND2-AS1 and miR-146. (**E**) The relative activity of the miR-146 promoter in the indicated cells was determined by dual-luciferase assay. miR-146wt, miR-146 wild-type promoter. miR-146mut, miR-146 mutated promoter. *P<0.05, vs. control, n=3. #*P*<0.05, vs. si-NC, n=3. (**F**) The expression of miR-146 wt or miR-146mut in 5637 cells expressing HAND2-AS1 or si-HAND2-AS1 was accessed by qRT-PCR. *P<0.05, vs. control, n=3. #*P*<0.05, vs. si-NC, n=3.

**Additional file 5: Fig. S4**. The overexpression of miR-146 promotes cell proliferation by targeting RARB. (**A**,** B**) The expression of RARB in cancer tissues and the corresponding adjacent tissues was determined by immunohistochemical staining and qRT-PCR, respectively. *P<0.05 vs. adjacent tissues. adj, adjacent tissues; can, cancer tissues. (**C**) The relationship between RARB and HAND2-AS1 expression in 32 pairs of bladder cancer tissues. (**D**) Left panel, schematic of the predicted binding sites of miR-146 and RARB; Right panel, the relative activity of the RARB promoter was determined by dual-luciferase assay. RARB, RARB wild type 3-’UTR; RARB Mut, RARB mutated 3-’UTR; miR-146 in, miR-146 inhibitor. **P<0.01, vs. scramble RNA, n=3. (**E**) The expression of RARB or miR-146 in the indicated cells was analyzed by qRT-PCR. *P<0.05, vs. scrambled RNA, n=3. Scr, scrambled RNA. (*F*) The expression of RARB in the indicated cells was analyzed by western blot. (**G**) The proliferation of 5637 and RT4 cells expressing miR-146in, sh-RARB or the combination was accessed by MTT assay. miR-146 in, miR-146 inhibitor. sh-RARB, shRNA targeting RARB. *P<0.05, vs. control, n=3. Scr, scramble RNA.

**Additional file 6: Fig. S5**. The overexpression of lncRNA HAND2-AS1 attenuates cell proliferation and enhances apoptosis by releasing RARB from miR-146. (**A**) The proliferation of the indicated cells was accessed by MTT assay. *P<0.05, vs. control, n=3. (**B**) The apoptosis of the indicated cells was detected by FITC-PI stain, followed by flow cytometry analysis. Representative images of three independent experiments were shown. *P<0.05 vs. vector. ns, no significance. (**C**) The expression of HAND2-AS1, miR-146, RARB, and Caspase 3 in the indicated cells were measured by qRT-PCR. *P<0.05 vs. control, n=3. ns, no significance. (**D**) The expression of HAND2-AS1, miR-146, RARB, and Caspase 3 in the indicated cells were measured by western blot.

**Additional file 7: Fig. S6**. The overexpression of lncRNA HAND2-AS1 suppresses tumor growth in 5637 human bladder cancer mouse models. (**A**) Tumor growth curves of xenografts for four weeks. *P<0.05; ns, no significance, vs. vector, 6 mice per group. (**B**) The median weights of tumors per group. *P<0.05; ns, no significance, vs. control, 6 mice per group. (**C**) The representative images of gross examination in each group were shown. (**D**) The expression of the indicated protein in tumor models was determined by western blot. (**E**) The expression of HAND2-AS1, miR-146, RARB, and Caspase 3 in tumors was determined by qRT-PCR. *P<0.05 vs. control, n=6.

## Data Availability

All data are included in the article, and all data obtained from RNA microarray is available in Gene Expression Omnibus database. The accession number is GSE140584, GSE140585 and GSE140587.

## Abbreviations

lncRNA: Long noncoding RNA
miRNA: MicroRNA
HAND2-AS1: HAND2 antisense RNA 1
RARB: Retinoic acid receptor-β
CDKN1A: Cyclin-dependent kinase inhibitor 1A
3'UTR: 3' Untranslational region
